# Effect of 3-nitropropionic acid inducing oxidative stress and apoptosis of granulosa cells in geese

**DOI:** 10.1042/BSR20180274

**Published:** 2018-09-12

**Authors:** Bo Kang, Xinxing Wang, Qilin Xu, Yongsheng Wu, Xiaohui Si, Dongmei Jiang

**Affiliations:** 1 College of Animal Science and Technology, Sichuan Agricultural University, Chengdu 611130, People’s Republic of China; 2 Institute of Animal Science, Chengdu Academy of Agriculture and Forestry Sciences, Chengdu, People’s Republic of China

**Keywords:** apoptosis, ferritin heavy chain, granulosa cell, oxidative stress, 3-nitropropionic acid

## Abstract

The mechanism of action by which oxidative stress induces granulosa cell apoptosis, which plays a vital role in initiating follicular atresia, is not well understood. In the present study, the effect of 3-nitropropionic acid (3-NPA) on oxidative stress and apoptosis in granulosa cells in geese was investigated. Our results showed that treatment with 3-NPA at 5.0 mmol/l for 24 h increased intracellular reactive oxygen species (ROS) production by 25.4% and decreased granulosa cell viability by 45.5% (*P*<0.05). Catalase and glutathione peroxidase gene expression levels in granulosa cells treated with 3-NPA were 1.32- and 0.49-fold compared with those of the control cells, respectively (*P* <0.05). A significant decrease in the expression level of B-cell lymphoma 2 (Bcl-2) protein and remarkable increases in the levels of Bax, p53 and cleaved-Caspase 3 proteins and the ratio of Bax/Bcl-2 expression in granulosa cells treated with 3-NPA were observed (*P*<0.05). Furthermore, a 38.43% increase in the percentage of early apoptotic cells was also observed in granulosa cells treated with 3-NPA (*P*<0.05). Moreover, the expression levels of *NF-κB, Nrf2, Fhc, Hspa2* and *Ho-1* in granulosa cells treated with 3-NPA were elevated 4.36-, 1.63-, 3.62-, 27.54- and 10.48-fold compared with those of the control cells (*P*<0.05), respectively. In conclusion, the present study demonstrates that treatment with 3-NPA induces ROS production and apoptosis and inhibits the viability of granulosa cells in geese. Furthermore, 3-NPA triggers increases in the expression of cleaved-Caspase 3 protein and the ratio of Bax/Bcl-2 expression, and induces the early apoptosis of granulosa cells.

## Introduction

Endogenous reactive oxygen species (ROS) play vital roles in signaling pathways including cell growth, metabolism, differentiation and apoptosis [1,2]. Excess ROS production causes lipid peroxidation and DNA damage, thereby inducing cell death [3,4]. Several studies have suggested that numerous ROS are produced by the ovaries in female animals during folliculogenesis and ovulation [5,6]. Granulosa cells, which surround oocytes in ovaries, play a pivotal role in follicular development, ovulation, atresia and steroidogenesis [7,8]. It is well known that oxidative stress induces granulosa cell apoptosis, which plays a vital role in initiating follicular atresia [9–11]. However, an understanding of these mechanisms is limited and remains to be defined.

The expression of genes related to inflammatory and oxidative stress can be rapidly activated by nuclear factor kappa-light-chain-enhancer of activated B cells (NF-κB). In addition, nuclear factor (erythroid-derived 2)-like 2 (Nrf2) is one of the transcription factors mediating antioxidant enzyme expression. Both NF-κB and Nrf2 are known to simultaneously initiate certain cellular responses to oxidative stress and are regarded as antioxidant response master switches in mammals [12–14]. Ferritin heavy chain (FHC) is a downstream target protein of both Nrf2 and NF-κB in mammals [15,16]. Yang et al*.* [17] suggested that FHC might be involved in regulating the ovulation of ovarian follicles and egg production in hens. Furthermore, FHC expression levels were greater in postovulatory and atresia follicles compared with those in the developing follicles [18]. These results indicated that FHC might regulate female reproduction through modulating follicular atresia and ovulation in birds.

3-Nitropropionic acid (3-NPA) irreversibly inhibits the activity of succinate dehydrogenase and promotes ROS formation, thereby inducing oxidative stress [13,19]. Several studies have suggested that 3-NPA significantly increases ROS production in granulosa cells and ovaries and then induces ovarian oxidative damage in mammals [20,21]. However, there are no data regarding the effect of 3-NPA on oxidative stress and apoptosis in granulosa cells in avian species.

In the present study, granulosa cells from geese were incubated in a cell culture medium supplemented with 3-NPA, and ROS production and the expression levels of genes related to cell proliferation, apoptosis and oxidative stress were evaluated, as well as the levels of the apoptosis-related proteins. The results showed that treatment with 3-NPA induced ROS production and apoptosis and inhibited the viability of granulosa cells in geese. Furthermore, 3-NPA triggered increases in the expression of cleaved-Caspase 3 protein and the ratio of Bax/Bcl-2 expression, and induced the early apoptosis of granulosa cells.

## Materials and methods

### Geese and primary granulosa cells

The Sichuan white goose care and use protocols were approved by the Animal Ethics Committee of the College of Animal Science and Technology at Sichuan Agricultural University. Female laying geese at the age of 7 months were killed by cervical dislocation. Follicle tissues and primary granulosa cells were quickly removed and processed as previously described [8,22]. In brief, granulosa cells were cultured in a DMEM/F12 medium supplemented with 3.0% FBS and 100 U/ml of penicillin/streptomycin in a humidified incubator at 37°C and 5.0% CO_2_. The granulosa cells were plated in 12-well plates at a concentration of 1.0 × 10^5^ cells/ml.

### Incubation and viability assay of primary granulosa cells

3-NPA was dissolved in phosphate buffer saline (PBS). Goose primary granulosa cells were cultured for 24 h *in vitro* and treated with various concentrations (0.1–20.0 mmol/l) of 3-NPA for another 24 h. Control granulosa cells were exposed to an equal volume of PBS. The viability of the granulosa cells was measured by the MTT method. Briefly, cells were plated at a density of 1.0 × 10^4^ cells/well in 96-well plates. After attachment, the cells were treated with 3-NPA in 0.1–20.0 mmol/l for 24 h. Then, the MTT solution dissolved in PBS at a final concentration of 0.5 mg/ml was added to each well, and the plates were incubated for another 4 h. The purple-blue MTT formazan precipitate was dissolved in 150.0 μl of dimethyl sulfoxide. Subsequently, the optical density (OD) at 490 nm was measured using a spectrophotometer (Thermo Fisher Scientific, U.S.A.). The percentage of cell viability was calculated as OD_3-NPA_/OD_Control_ × 100%.

### Measurement of intracellular ROS

ROS levels in granulosa cells treated with 3-NPA were measured using an ROS Assay Kit (Beyotime, China). Briefly, cells were seeded at a density of 1.0 × 10^4^ cells/well in a 96-well plate. Next, granulosa cells were treated with 3-NPA at 5.0 mmol/l, the medium in each well was removed, and 10.0 μmol/l 2,7-dichlorodihydrofluorescein diacetate (DCFH-DA) was added to the plate, which was then incubated for 20 min at 37°C in a humidified 5.0% CO_2_ atmosphere. Extracellular DCFH-DA was subsequently removed by washing with PBS three times. The fluorescence intensity was determined with a fluorescence spectrophotometer (Thermo Fisher Scientific, U.S.A.), using 488 and 525 nm as the excitation and emission wavelengths respectively. The fluorescence image was captured with confocal laser scanning microscope (Olympus, Japan). Quantitative data of fluorescence intensity were standardized by dividing each value by the average value of the control group in each experiment. The results are representative of three independent experiments.

### Quantitative real-time PCR

RNA isolation and cDNA synthesis in granulosa cells were performed using the TRIzol reagent and PrimeScript^®^RT reagent Kit (Takara Bio Inc., China), according to the manufacturer instructions. The primer sets used are described in Table 1. The quantitative real-time PCR (qRT-PCR) was carried out in a 10.0 μl reaction using iTaq^TM^ SYBR^®^ Green Supermix (Bio-Rad, U.S.A.). The reaction containing 5.0 μl of SYBR^®^ Green Supermix, 4.1 μl of RNase-free water, 0.5 μl of cDNA and 0.2 μl of each of the primers was performed as follows: 95°C for 3 min; 40 cycles of 95°C for 10 s; 55–65°C (according to Table 1) for 30 s; and 72°C for 30 s, followed by measuring the melting curves. The qRT-PCR was carried out in a 96-well iCycle CFX96 (Bio-Rad, U.S.A.). The 2^–∆∆C_t_^ method was employed to analyze the mRNA expression levels of genes. *Gapdh* was used as the reference gene. The relative quantitation of gene expression was performed in three replicates for each sample.

**Table 1:** Primers used in the present study

Primers	Sequence (5′-3′)	Size (bp)	*T*_m_ (°C)
*Cat*	F: ATACAGTTCGTGACCCTCG	188	56
	R: CCAGAAGTCCCATACCAT		
*Sod*	F: AAATGGGTGTACCAGCGCAG	138	57
	R:TCTTCTATTTCTACTTCTGCCACTCC		
*Gpx*	F: GCAAGGGGTACAAGCCCAACT	149	59
	R: GATGATGTACTGCGGGTTGGTC		
*Ccnd1*	F:TGTTTACGAGCCTGCCAAGAA	109	55
	R: CTGCTTCGTCCTCTACAGTCTTTG		
*Pcna*	F: AGAAATGAATGAGCCAGTCCAGC	178	55
	R: TTCAATCTTTGGAGCCAGGTAGT		
*Bcl-2*	F: GATGCCTTCGTGGAGTTGTATG	98	60
	R: GCTCCCACCAGAACCAAAC		
*p53*	F: GCCCAACCTCGCTAAGAA	197	63
	R: CAACCACCATCCCTGACG		
*Caspase 8*	F: GGTGTCGCAGTTCAGGTA	127	57
	R: CATTGTAGTTTCAGGGCTT		
*Caspase 9*	F: TTCCAGGCTCTGTCGGGTAA	150	64
	R: GTCCAGCGTTTCCACATACCA		
*Caspase 3*	F: CTGGTATTGAGGCAGACAGTGG	158	60
	R: CAGCACCCTACACAGAGACTGAA		
*NF-κB*	F: TCAACGCAGGACCTAAAGACAT	162	56
	R: GCAGATAGCCAAGTTCAGGATG		
*Nrf2*	F: CGCCTTGAAGCTCATCTCAC	176	55
	R: TTCTTGCCTCTCCTGCGTAT		
*Fhc*	F: CGCCAGAACTACCACCAGG	123	63
	R: TTTCAGAGCCACATCATCCC		
*Hspa2*	F: GCTGGGCAAGTTTGATCTAA	238	58
	R: ATCTCTGTTGGCTTCGTCCTC		
*Ho-1*	F: TGCCTACACTCGCTATCTGG	183	60
	R: AGGTCCATCTCAAGGGCATT		
*Gapdh*	F: GTGGTGCAAGAGGCATTGCTGAC	86	65
	R: GCTGATGCTCCCATGTTCGTGAT		

### Western blot

Granulosa cells were incubated with 3-NPA at 5.0 mmol/l for 24 h and then were harvested. The total protein was extracted using RIPA Lysis Buffer and 10% phenylmethanesulfonyl fluoride (Beyotime, China). Protein concentration was determined by using a BCA Protein Assay Kit (Beyotime, China). Approximately, the same amount of protein was separated using 10–12% SDS-PAGE, transferred electrophoretically onto the polyvinylidene membrane (Bio-Rad) and blocked with 5% nonfat dry milk. The primary antibodies used in the present study were anti-Caspase 3 (CST, U.S.A.), anti-Bcl-2 (Wanlei Biotechnology, China), anti-p53 (Wanlei Biotechnology, China), anti-Bax (Bioss Biotechnology, China), anti-β-actin (TransGen Biotechnology, China). The membrane was incubated with the primary antibody solution overnight at 4°C, and then washed four times with the TBST (TBS, 0.1% Tween 20). The corresponding secondary antibody (1:5000) was added and incubated at room temperature for 1 h. The protein bands were visualized by using the BeyoECL Plus (a chemiluminescence reaction; Beyotime, China) in an Image Lab software (Bio-Rad, U.S.A.). The bands were quantified using an ImageJ software (NIH, U.S.A.).

### Flow cytometric analysis

Cell apoptosis was determined by flow cytometry (BD Biosciences, U.S.A.) using an Annexin V-fluorescein isothiocyanate (FITC)/propidium iodide (PI) kit (BD Biosciences, U.S.A.), according to the manufacturer’s protocol. Briefly, Granulosa cells were seeded in 12-well plates with a density of 1 × 10^6^ cells/well for 24 h and then treated with 3-NPA at 5.0 mmol/l for another 24 h. Granulosa cells were harvested and washed twice with cold PBS, and labeled with Annexin V-FITC and PI for 15 min at 25°C in the dark in binding buffer. Fluorescence intensity of granulosa cells was detected by flow cytometry within 1 h. The analysis was replicated thrice and the apoptosis rate (%) for each treatment was obtained.

### Statistical analyses

All data were statistically analyzed by one-way analysis of variance using SAS 9.0 (SAS Institute Inc., U.S.A.). Statistically significant results were further analyzed by Duncan’s multiple range test. Data are all presented as the mean ±SEM. A *P* value of <0.05 was considered significant.

## Results

### 3-NPA reduced granulosa cell viability

Compared with control cells, no visible morphological changes were detected in granulosa cells exposed to 0.1–5.0 mmol/l 3-NPA for 24 h. However, with increased 3-NPA concentration to 0.1–5.0 mmol/l, granulosa cell viability decreased gradually (Figure 1). The viability of granulosa cells treated with 3-NPA at 5.0 mmol/l for 24 h decreased by 45.5% compared with that of the control cells (*P*<0.05). With further increases of the 3-NPA concentration, the occurrence of granulosa cell death increased sharply. In the following study, 3-NPA at 5.0 mmol/l was employed to treat granulosa cells.

**Figure 1:** Effect of 3-NPA on granulosa cell viability The viability of granulosa cells exposed to 3-NPA (0.1–20.0 mmol/l) for 24 h was measured by MTT and presented as a percentage of the control value (*n*=8). Control granulosa cells were treated with PBS only. All data are presented as the mean ± SEM. *P<0.05 compared with the control.

### 3-NPA increased ROS production and *Cat* expression and decreased *Gpx* expression

ROS play a key role in cell apoptosis. Therefore, the effect of 3-NPA on ROS generation in granulosa cells was determined. The fluorescence intensity of granulosa cells reflects the level of ROS production. The results showed that 3-NPA increased markedly the fluorescence intensity of granulosa cells compared with that of the control cells (Figure 2A), suggesting that 3-NPA induced the generation of intracellular ROS. Furthermore, a 25.4% increase in ROS production was recorded in granulosa cells exposed to 3-NPA at 5.0 mmol/l for 24 h (*P*<0.05; Figure 2B). The levels of catalase (CAT) and glutathione peroxidase (GPX) in granulosa cells treated with 3-NPA were 1.32- and 0.49-fold compared with those of the control cells, respectively (*P*<0.05), while superoxide dismutase (SOD) expression levels were not significantly different in granulosa cells exposed to 3-NPA compared with those of the control cells (*P*>0.05; Figure 2C).

**Figure 2:** Level of ROS production and *Cat, Sod* and *Gpx* mRNA expression in granulosa cells Granulosa cells were treated with 3-NPA at 5.0 mmol/l for 24 h. (**A**) Representative fluorescence image of ROS production visualized using DCFH-DA by confocal laser scanning microscope; scale bar, 25 μm. (**B**) Level of ROS production determined using DCFH-DA in granulosa cells. (**C**) Levels of *Cat, Sod* and *Gpx* mRNA expression. Data are presented as the mean ± SEM. *P<0.05 compared with the respective control.

### 3-NPA regulated the transcription of genes related to cell proliferation and apoptosis

To explore the effect of 3-NPA on cell proliferation and apoptosis, the mRNA expression levels of cyclin D1 (*Ccnd1*), *Pcna, Bcl-2, p53* and *Caspase 3, Caspase 8* and *Caspase 9* in granulosa cells treated with 3-NPA at 5.0 mmol/l were measured (Figure 3). The expression levels of *Pcna, p53* and *Caspase 8* in granulosa cells exposed to 5.0 mmol/l 3-NPA were 0.56-, 0.39- and 0.51-fold compared with those of the control cells (*P*<0.05), respectively. The mRNA expression levels of *Bcl-2* and *Caspase 3* in granulosa cells exposed to 5.0 mmol/l 3-NPA were 5.93- and 1.91-fold compared with those of the control (*P*<0.05), respectively.

**Figure 3:** Effect of 3-NPA on cell proliferation and apoptosis gene expression Data are presented as the mean ± SEM. Bars with the same letter are not significantly different (*P*<0.05). *P<0.05 compared with the respective control.

### 3-NPA elevated the expression of Bax, p53 and cleaved-Caspase 3 proteins and decreased Bcl-2 expression

To further investigate the effect of 3-NPA on granulosa cell apoptosis, the levels of the apoptosis-related proteins such as Bcl-2, Bax, p53, Caspase 3 and cleaved-Caspase 3 were detected using Western blot. The results showed a significant decrease in the expression level of Bcl-2 protein and a remarkable increase in the levels of Bax, p53 and cleaved-Caspase 3 proteins after 24 h of treatment with 3-NPA at 5.0 mmol/l (*P*<0.05; Figure 4A, B). Meanwhile, the ratio of Bax/Bcl-2 in granulosa cells exposed to 3-NPA was significantly higher than that of the control cells (*P*<0.05) and was increased by 3.59-fold compared with that of the control cells (Figure 4C).

**Figure 4:** Expression of proteins related to apoptosis Granulosa cells were treated with 3-NPA at 5.0 mmol/l for 24 h. (**A**) The expression of Bcl-2, Bax, p53, Caspase 3, cleaved-Caspase 3 and β-actin in granulosa cells was determined by Western blot. (**B**) The expression of Bcl-2, Bax, p53 and cleaved-Caspase 3 was quantified by densitometry, and data were normalized to β-actin. (**C**) Ratios of Bax/Bcl-2 expression. Data are presented as the mean ± SEM. *P<0.05 compared with the respective control.

### 3-NPA induced early apoptosis in granulosa cells

Flow cytometry using Annexin V-FITC/PI was further employed to confirm the apoptosis-inducing effect of 3-NPA on granulosa cells (Figure 5). Significant increase of early apoptosis was observed in granulosa cells treated with 3-NPA at 5.0 mmol/l for 24 h (*P*<0.05). A 38.43% increase in the percentage of early apoptotic cells was recorded in the granulosa cells treated with 3-NPA. It could be suggested that 3-NPA at 5.0 mmol/l for 24 h induced early apoptosis of granulosa cells. However, the percentage of late apoptotic cells in the granulosa cells treated with 3-NPA was not significantly different compared with that of the control cells (*P*>0.05).

**Figure 5:** Flow cytometry analysis of granulosa cell apoptosis by double staining with Annexin V-FITC and propidium iodide (PI) Granulosa cells were treated with 3-NPA at 5.0 mmol/l for 24 h. Data are presented as the mean ± SEM. *P<0.05 compared with the respective control; LL, living cells An-/PI-; LR, early apoptotic cells An+/PI-; UR, late apoptotic cells An+/PI+; UL, necrotic cells An-/PI+.

### 3-NPA up-regulated *NF-κB, Nrf2, Fhc, Hspa2* and *Ho-1* mRNA expression

To uncover the effect of 3-NPA on the expression of oxidative stress downstream target genes in granulosa cells in geese, expression levels of key genes related to the NF-κB and Nrf2 pathways were investigated (Figure 6). As expected, the mRNA expression levels of *NF-κB, Nrf2, Fhc*, heat shock protein family A (Hsp70) member 2 (*Hspa2*; encoding a heat shock protein) and *Ho-1* in granulosa cells exposed to 5.0 mmol/l 3-NPA were significantly higher than those of the control cells (*P*<0.05) and were increased by 4.36-, 1.63-, 3.62-, 27.54- and 10.48-fold compared with those of the control cells, respectively.

**Figure 6:** Effect of 3-NPA on expression levels of genes related to the NF-κB and Nrf2 pathways Data are presented as the mean ± SEM. Bars with the same letter are not significantly different (*P*<0.05). *P<0.05 compared with the respective control.

## Discussion

ROS at physiological levels is necessary for maintaining follicular and ovarian functions. However, excessive ROS generation in follicles induces oxidative stress and initiates granulosa cell apoptosis and follicular atresia [23,24]. 3-NPA inhibits the succinate dehydrogenase catalytic site, blocks the electron transport chain and the Krebs cycle, decreases ATP synthesis and promotes ROS formation [25]. In the present study, ROS production increased by 25.4% and granulosa cell viability decreased simultaneously by 45.5% in granulosa cells exposed to 3-NPA at 5.0 mmol/l. Furthermore, significant increase in the fluorescence intensity of granulosa cells treated with 3-NPA also indicated that 3-NPA increased ROS products. This result is consistent with a previous study in which Zhang et al. [26] reported that 3-NPA increased ROS generation in mouse ovaries. These findings imply that 3-NPA promotes ROS generation and induces oxidative stress in tissues and cells in both mammals and birds. SOD can rapidly convert O_2_^−^ to H_2_O_2_, and CAT and GPX catalyze the decomposition of H_2_O_2_ to water. Mandavilli et al*.* [27] reported that 3-NPA treatment caused a dose-dependent rapid increase in H_2_O_2_ production in rat pheochromocytoma cells. Our results showed that treatment with 5.0 mmol/l 3-NPA significantly elevated the mRNA expression level of *Cat* and obviously decreased the mRNA expression level of *Gpx* in goose granulosa cells. Simultaneously, no significant difference in *Sod* expression level was observed. These results indicated that ROS products induced by 3-NPA modulated the levels of *Cat* and *Gpx* mRNA expression in granulosa cells. Additionally, one study reported an inconsistent result in which the mRNA expression levels of *Sod* and *Gpx* increased significantly in granulosa cells in mice injected intraperitoneally with 12.5 mg/kg 3-NPA for 7 days, while no significant change in the expression of *Cat* was observed [20]. This finding indicates that the effect of 3-NPA on antioxidant enzyme gene expression in granulosa cells may be different *in vivo* and *in vitro*.

Proliferating cell nuclear antigen (PCNA), a marker of cell proliferation, is highly expressed in proliferating cells. The tumor suppressor p53 plays important roles in regulating intracellular redox [28,29]. 3-NPA can increase the mouse ovarian ROS levels and up-regulate the apoptosis-related gene *Caspase 3* in mouse granulosa cells [26]. Our results showed that in goose granulosa cells, treatment with 3-NPA at 5.0 mmol/l down-regulated the mRNA expression of *Pcna* and *p53*, while it up-regulated *Caspase 3* mRNA expression. It is plausible that the diminished proliferative and augmented apoptosis caused by the transient oxidative stress induced by 3-NPA may contribute to the inhibition of granulosa cell viability in geese [30]. The anti-apoptotic protein Bcl-2 inhibits cytochrome *c* release and Caspase 3 activation and thus functions as an antioxidant to prevent apoptosis [31]. Elevated levels of ROS and *Bcl-2* mRNA expression were observed in granulosa cells exposed to 3-NPA in the present experiment. This finding is consistent with the hypothesis that ROS generation is the primary event in 3-NPA toxicity and that Bcl-2 protects cells from 3-NPA toxicity by preventing mitochondrial DNA damage [27]. However, in granulosa cells treated with 3-NPA at 5.0 mmol/l, the reason why the mRNA expression level of the initiator *Caspase 8* decreased but that of *Caspase 9* showed no significant changes remains to be investigated.

As mentioned above, excessive ROS generation in follicles induces oxidative stress and initiates granulosa cell apoptosis. Many studies have emphasized the relationship between mitochondrial dysfunction and cell apoptosis. In the present study, cleaved-Caspase 3 and pro-apoptotic Bax were significantly up-regulated in granulosa cells treated with 3-NPA, while anti-apoptotic Bcl-2 was correspondingly down-regulated. Furthermore, remarkable increases in both the ratio of Bax/Bcl-2 expression and the percentage of early apoptotic cells were also observed. Bax forms ion channels directly causing mitochondria to release cytochrome *c* and then activates Caspase-3, which induces apoptosis in the end [32,33]. Therefore, all these findings demonstrated that 3-NPA induced mitochondrial apoptosis in granulosa cells. The tumor suppressor p53 plays key and complex roles in cellular responses to oxidative stresses. In response to low levels of oxidative stresses, p53 plays primarily antioxidant roles [34]; in response to high levels of oxidative stresses, p53 exhibits pro-oxidative activities [35,36]. Our results revealed that treatment with 3-NPA elevated remarkably the expression of p53 protein, while the mRNA level of p53 was regulated by 3-NPA accordingly. Further study elucidating the effect of 3-NPA on the expression of p53 protein and gene in granulosa cells should be carried out. ROS are generated by many cellular processes as part of cellular signaling events. Both NF-κB and Nrf2 function as key antioxidant transcription factors in response to ROS. A number of studies have suggested that NF-κB and Nrf2 signaling pathways are involved in regulating oxidative stress [37–39]. Zhang et al. [40] suggested that phosphorylated NF-κB expression increased in a dose- and time-dependent manner in granulosa cells treated with H_2_O_2_. 3-NPA treatment up-regulated the levels of NF-κB protein and *Nrf2* gene expression in the mouse striatum [41]. In agreement with these findings, our data showed that increased intracellular ROS production induced by 3-NPA up-regulated *NF-κB* and *Nrf2* mRNA expression in goose granulosa cells. FHC up-regulation by NF-κB inhibits TNF-α-induced apoptosis by suppressing ROS [16]. Nrf2 can be activated by ROS and thus binds to the antioxidant response element of *Fhc*, which in turn induces FHC antioxidant activity [15]. In the present study, the finding that 3-NPA treatment significantly increased *Fhc* expression in granulosa cells confirms that FHC has an important antioxidant action in granulosa cells. Therefore, it is not surprising that ROS through the NF-κB and Nrf2 pathways up-regulates the mRNA expression of *Fhc* to attenuate ROS toxicity. Taken together, *Fhc* mRNA expression up-regulation by 3-NPA indicated that FHC might be essential for modulating the response of granulosa cells to oxidative stress induced by 3-NPA through the NF-κB and Nrf2 antioxidant pathways, although the exact mechanism remains to be investigated. Given that birds only express FHC but lacks an intact ferritin light chain [42], a suitable experimental setting to investigate the mechanism of FHC-mediating oxidative stress induced by 3-NPA should be carried out in a future study. ROS disrupts Keap1–Nrf2 interactions and thus promotes Nrf2 activation. Nrf2 binds to antioxidant response element and induces the expression of numerous antioxidants, including heme oxygenase 1 (HO-1) and heat shock proteins [15,43,44]. In the present study, treatment with 3-NPA significantly increased the mRNA expression level of *Ho-1* and *Hspa2*. In agreement with our findings, several studies have suggested that ROS elevates the mRNA expression of *Ho-1* and *Hspa2* in mice [15,41,45].

## Conclusions

The present study demonstrates that treatment with 3-NPA induces ROS production and apoptosis and inhibits the viability of granulosa cells in geese. Furthermore, 3-NPA triggers increases in the expression of cleaved-Caspase 3 protein and the ratio of Bax/Bcl-2 expression, and induces the early apoptosis of granulosa cells. However, additional studies are required to investigate the true role of FHC in modulating the response of granulosa cells to oxidative stress induced by 3-NPA through the NF-κB and Nrf2 antioxidant pathways.

## Abbreviations

3-NPA: 3-nitropropionic acid
Bcl-2: B-cell lymphoma 2
CCND1: cyclin D1
FHC: ferritin heavy chain
HO-1: heme oxygenase 1
HSPA2: heat shock protein family A (Hsp70) member 2
NF-κB: nuclear factor kappa-light-chain-enhancer of activated B cells
NRF2: nuclear factor (erythroid-derived 2)-like 2
PCNA: proliferating cell nuclear antigen
ROS: reactive oxygen species
TNF-α: tumor necrosis factor α
